# Fisheries and Marine Animal Populations: Learning from the Long Term

**DOI:** 10.1371/journal.pone.0016011

**Published:** 2011-01-07

**Authors:** David J. Starkey, Tim D. Smith, Michaela Barnard

**Affiliations:** 1 Department of History, University of Hull, Hull, United Kingdom; 2 History of Marine Animal Populations, Redding, California, United States of America; University of Western Ontario, Canada

The articles that comprise the HMAP Collection are products of the History of Marine Animal Populations (HMAP) project. This is an international, multidisciplinary initiative, the overarching aim of which is to improve knowledge and understanding of the long-term interaction of humankind with the marine environment. HMAP endeavours to attain this goal in three principal ways. First, a concerted effort is being made to embed the approaches and methods developed by HMAP into the institutional fabric of the universities that are hosting the project. This connects closely with the second strand of the scheme, which is designed to develop the parallel disciplines of historical marine ecology and marine environmental history through the sponsorship of graduate studentships, workshops, summer schools, conferences and the dissemination of research outputs. The third activity is the co-ordination of a research programme embracing the efforts of over 100 scientists in 18 countries working in teams tasked with investigating 12 regionally-specific, two thematic and two global taxon-specific case studies [www.hmapcoml.org/projects]. HMAP has progressed fruitfully in all three respects since its inception in 2000. It has established centres at the universities of New Hampshire (USA), Roskilde (Denmark), Hull (UK), Murdoch (Australia) and Trinity College Dublin (Ireland), where faculty members – some of whom might be cast as ‘HMAP graduates’ - are responsible for leading the project and cultivating its distinctive approach to marine environmental issues. Here, and at numerous other educational institutions, the curricula have been enriched by the introduction of programs of study that focus on the marine dimensions of historical ecology and environmental history. Such learning and teaching work is informed by research undertaken under the aegis of HMAP, which by 2009 had generated over 200 printed and online works [www.hmapcoml.org/publications], as well as a substantial web-based data store [1], an online atlas of fisheries in the case study areas [2] and an image gallery [3]. The articles in the HMAP Collection add to that output. Some were generated by scientists funded as part of the HMAP research effort, while others had their genesis in papers presented at ‘Oceans Past II: Multidisciplinary Perspectives on the History and Future of Marine Animal Populations’, an international conference convened by HMAP and hosted by the Aquatic Ecosystem Research Laboratory at the University of British Columbia in May 2009. The Collection testifies to the vitality of the HMAP approach to the dynamic interaction of humankind and the marine environment. This overview explains how that approach evolved, identifies the research issues that lie at its heart, and outlines some of the contributions to knowledge and understanding that HMAP research has yielded.

## Introduction

### The need for a long-term perspective

The History of Marine Animal Populations project was conceived in the late 1990s. It swiftly hatched into the historical component of the primarily science-based Census of Marine Life (CoML) program, which aims to assess and explain the diversity, distribution, and abundance of life in the oceans - past, present and future [4]. That a historical dimension was integral to the initial CoML research agenda indicates that the census-makers recognised how ‘a survey of contemporary marine life would have much more value if compared with historical information’ [5]. This recognition implied that significant explanatory insight could ensue from measuring the present state of ocean life against conditions in a ‘lost past’ that might to some extent be recovered through historical research into the efforts of humans to extract fish from the seas over the long term. In turn, such research promised to reveal the degree to which marine life now, and in the future, has been ‘influenced and cultured by the courage, ingenuity and folly of human endeavour’ in the past [5].

The integration of history into the science-driven CoML reflected developments in four disciplines - archaeology, history, biology and ecology - during the final third of the twentieth century. In essence, specialisation in these fields of enquiry led to the emergence of a number of sub-disciplines that converged in the 1990s to offer a multidisciplinary, or holistic, perspective on the long-term interaction of human and marine life. Since the 1960s, for instance, developments in archaeological science have given rise to paleoecology, archaeoichthyology and paleozoology. In one example of the fruits of these sub-disciplines, the preservation of fish scales in anaerobic bottom sediments off the coast of California enabled scientists to reconstruct 1600 years of pelagic abundances [6]–[8]. Paleozoologists likewise bridged the cultural divides of history and ecology during the 1990s by analysing fish remains from archaeological sites to understand better the diversity, distribution and abundance of species [9], [10]. Fish bones were also used to test the accuracy of climate models, some of which predict that air and sea temperatures will rise by approximately 3°C during the next 70–100 years. In order to understand some of the processes by which such global warming might affect marine fish species near Denmark, researchers investigated fish fauna deriving from one of the warmest prehistoric periods (the warm Atlantic period: ca. 7000–3900 BC). A total of 108,000 fish bones were identified, including those from species such as anchovy and black sea bream, which normally live in warmer, more southerly waters, like those of the Mediterranean. When temperatures cooled after the warm period ended, most of these species disappeared from the archaeological record, suggesting that local abundances declined [11]. However, since the early 1990s, many of these warm-water species have reappeared in waters around Denmark as temperatures have risen, suggesting that archaeological information can identify which species may become common if global warming occurs.

Specialist sub-disciplines have evolved within the history discipline since the 1960s. Environmental history was one of these off-shoots, sprouting in the USA during the 1970s and growing ever since, a pattern evident, albeit a little later, in Europe, Asia, Australia and, despite institutional problems, South America and Africa. However, the focus of the pioneering American environmental historians was strongly on human agency and perception, with ecological factors rarely afforded an explanatory role. Moreover, the sub-discipline developed out of a strongly narrative and qualitative approach to history that had little rapport with the quantitative approach of ecologists. The focus was very much on frontier cultures of the prairies, bushlands, savannahs and steppes, while the oceans were largely disregarded [12]. On the other hand, maritime historians - another emerging specialist group – generally adopted an economic and social approach, and were so preoccupied with naval and shipping themes that they paid little heed to environmental issues. There were a few fisheries historians, but they often found their subject of marginal interest to mainstream historians and were rather fuzzy about the ecological facets of fishing, knowing they could not be neglected, but making little effort to understand them. Published overviews of fisheries were rare and generally adopted a national, regional or port perspective, while environmental considerations were incidental at best [13]. It was not until 1995 that the North Atlantic Fisheries History Association was established, but even then few of its outputs dealt with the impact of harvesting on the seas [14]–[17]. Signs of change were nevertheless evident as the twentieth century drew to a close. In 1995, scholars from the natural and social sciences, as well as the humanities, participated in a conference convened at the Memorial University of Newfoundland with the aim of assessing the scale, impact and management of fishing effort in the North Atlantic region since c.1500 [18]. Three years later, Holm and Starkey reported the results of ‘Fishing Matters’, a workshop held in Denmark that brought together historians, social scientists, biologists, oceanographers and fisheries managers to examine multidisciplinary approaches to understanding the past and current scale and character of the fisheries [19]. On the shores of the North Pacific, Pauly, Pitcher and Presiloshot organised a meeting in 1998 aimed at mathematically reconstructing the state of the Strait of Georgia, off Vancouver Island. Participants were drawn from various backgrounds, their challenge being ‘to provide a vision for rebuilding the Strait's once abundant resources’ [19].

The interest of natural scientists in the fisheries dates back to the late nineteenth century, when governments began to address the question of fluctuations in catches, largely because the social and economic costs of this unpredictability were high. Two schools of thought emerged. Some scientists explained the often large fluctuations and long-term declines from a single species perspective. This simplicity allowed them to provide more concrete advice to fisheries managers. Other scientists, however, saw the problem as involving multiple interacting species, an ecological perspective that had its origins in a terrestrial setting, and was now applied to the sea [20]. These two perspectives initially developed concurrently, but by the 1920s they had separated into two distinct disciplines - fisheries biology and marine ecology [21], [22]. Whereas fisheries biologists increasingly focused on self-regulating population models that could be used as a basis for quantitative advice to fisheries managers, marine ecologists concentrated on biodiversity, food-webs and biological processes. For the fisheries biologists, the ultimate question was how to predict sustainable catch levels, but with any other human impacts left out. In contrast, the ultimate question for the marine ecologists was not what is in the sea for us, the humans, but how do we understand nature on its own, again with the humans left out. Nevertheless, both disciplines continued to share the assumption that equilibrium or steady-state models were sufficient because changes were expected to be followed by more or less rapid transitions to new equilibrium conditions. The history of fisheries and ecosystems could safely be ignored as the dynamics and new equilibrium states were determined primarily by current conditions. By the 1950s, however, it was becoming clear that ecosystems rarely remain steady for long, as ‘fluctuations lie in the very essence of the ecosystems and of every one of the … populations’ [23]. Fisheries biologists and marine ecologists, who had hitherto perceived little or no need to consider the history of the systems they were studying, were now challenged with the reality that equilibrium baseline conditions were difficult to define and that in any event present conditions were often strongly affected by earlier events.

Fisheries biologists began to recognize the need for a more historical perspective on some fisheries. Papers summarizing long-term landings were therefore published, especially for fisheries where management depended on the relationships between numbers of spawners and resulting number of recruits [24] or on estimates of maximum sustainable yield [25]. Long time series of landings for most fisheries, however, became unnecessary when management came increasingly to depend on virtual population analyses, as these calculations were only sensitive to the age structure of recent landings [22]. Another sign of this growing historical awareness was the recognition that some formerly important fishes no longer occurred in harvestable numbers, as Goode and Collins had demonstrated in the 1880s for Atlantic halibut in New England waters [26]. This was especially the case for whaling, where several populations of whales had nearly been exterminated in the nineteenth century. Because of the extreme levels of depletion of whales that had occurred, and because of the long lifespan of large whales, the effects of whaling even 100 years previously were important to an understanding of the current state of whale populations. Accordingly, by the mid-1980s, scientists were combing through nineteenth-century whaling logbooks for evidence of the scale and distribution of past catches [27].

A number of ecologists also made the historical turn. In 1995, Daniel Pauly observed that most equilibrium or steady-state models are based on a given dataset, often established by scientists within the last generation [28]. But what happens to the equilibrium models if older data are introduced? We cannot know from recent information the extent of the losses that have already happened. In a seminal study of the Caribbean ecosystem, J.C.B. Jackson made the scathing remark that the child assumes that the world as s/he sees it first is the natural condition of the world – and ecologists have often assumed that the natural or original condition is equal to the first scientific description of a phenomenon. His critique was set within an empirical study of the trade in Caribbean turtles that deployed evidence from eighteenth-century British colonial trade statistics to ascertain that hundreds of thousands of turtles were killed annually. This persuaded Jackson that the ecosystem of the Caribbean would have looked very different to the scenario that conservation biologists had supposed on the basis of information relating to the last couple of decades [29]. The lesson to ecologists of Jackson's historical analysis of Caribbean coral reefs was that textbook descriptions of reef ecosystems were limited by the fact that systematic descriptions by modern biologists only began in the 1950s. Jackson put the case squarely to the ecologists: they needed to turn to historical sources and rediscover the world. This argument was pressed home in 2001, when Jackson and his colleagues asserted that ‘more specific paleoecological, archaeological, and historical data should be obtained to refine the histories of specific ecosystems and as a tool for management’ [30]. Once more the scope of previous ecological and marine biological investigations was criticized on the grounds that ‘most ecological research is based on local field studies lasting only a few years and conducted sometime after the 1950s without longer term historical perspective’ [30].

With the long-term perspective finding favour in the marine sciences, and ecological approaches assuming more importance in the analyses of archaeologists and historians, a prospectus for a History of Marine Animal Populations project was issued in 1999 [19]. This received the backing of the Sloan Foundation and of the promoters of the CoML initiative, and a workshop was convened to scope the HMAP project.

### HMAP: parameters and key research questions

The initial phase of HMAP was characterized by discussions about the nature and scope of what was appropriate and possible historically and scientifically that would contribute to the present and future foci of the Census of Marine Life. These deliberations culminated in a workshop held in Denmark in February 2000, at which researchers from various disciplines involved in CoML sought to define and encourage what was quickly seen to be a necessary and needed expansion of both environmental history and historical ecology, as well as an important component of the Census. The meeting yielded an analytical framework, a set of hypotheses and an edited collection of papers [31].

It was agreed that the topical, spatial and temporal parameters of HMAP should be broad: that is, the project should investigate the impact of human activity on marine animal populations in the world's seas and oceans over the last 2,000 years. But four provisos were identified. First, much of what can be known about the history of marine animal populations relates to the ‘human edges’ of the ocean, the near shore and coastal waters where humans most directly interacted with the sea in the past – as a source of food, a means of transportation, a theatre of war and a recreational zone. Accordingly, most historical records concern such activities in this realm. Second, the research should focus on the human activity that has had the greatest impact on marine ecosystems over historic time, the commercial fisheries conducted on the human edges and (for certain species) in mid-oceanic waters. Third, in generating knowledge about the impact and significance of the commercial fisheries, it is inevitable that analyses will be skewed towards the extraction of large animals, notably whales, large fish (such as cod and bluefin tuna), and marketable smaller species (like herring), where the sheer size and/or commercial value of the organisms encouraged captors to create and maintain archival material. Fourth, moving from the unknown to the known history of the oceans requires that the approaches and methods of archaeology, history, biology and ecology be deployed in a truly multidisciplinary way.

A preliminary set of hypotheses was also formulated at the 2000 workshop (http://hmapcoml.org/documents/Hypotheses.pdf). From this, four broad research questions were devised:

- How have the diversity, distribution, and abundance of marine animal populations altered over the last 2,000 years?
- Which factors have forced or influenced changes in the diversity, distribution, and abundance of marine animal populations?
- What has been the anthropogenic and biological significance of changes in marine animal populations?
- By what processes have marine ecosystems interacted with human societies?

The workshop recognised that a range of practical factors would necessarily restrict the research to sub-projects selected according to their intellectual rigour, viability in terms of primary sources, cost and personnel, and fit with the project's key research questions. Henceforth, the HMAP research effort progressed on a case study basis, with a core of initial studies augmented by later investigations that extended knowledge and understanding of past ocean life over time and space. The HMAP Collection indicates that this process of knowledge accretion continues unabated.

## Results and Discussion

### The HMAP Collection in an HMAP research context

The HMAP project has generated a sizeable volume of research products. Yet the fact that over 60% of the papers presented to the Oceans Past II Conference in May 2009 were delivered by researchers who had not previously been engaged in the project suggests that the HMAP approach is being adopted by a growing number of scientists and historians. The composition of the conference programme also implied that new subjects are being investigated, while the initial HMAP studies continue to stimulate research. The HMAP Collection confirms these impressions, for it comprises papers that in different ways extend the scope of HMAP, and papers that build upon established HMAP themes and approaches.

Two papers in the HMAP Collection focus on the Northern Adriatic Sea. In one, Shimrit Perkol-Finkel and Laura Airoldi push the frontiers of HMAP research into the sub-tidal zone in their study of habitat resilience in algal forests of the Adriatic coastline [32]. As they point out, habitat loss is often caused by gradual, long-term changes that impair the ability of natural ecosystems to absorb and recover from natural and human influences. Deploying a combination of historical data, and quantitative *in situ* observations of natural recruitment patterns, the authors argue that recent contractions in forest areas along the urbanized coasts of the north Adriatic Sea were triggered by accelerating cumulative impacts of natural- and human-induced habitat instability, exacerbated by an increase in the occurrence and severity of storms. Having examined the prospects for restoring such diminished habitats, Perkol-Finkel and Airoldi emphasize that better protection of natural habitats is required, as the restoration of pre-degradation environmental conditions, if possible, is often not cost-effective. In the second Adriatic paper, Tomaso Fortibuoni, Simone Libralato, Saša Raicevich, Otello Giovanardi and Cosimo Solidoro assess the utility of qualitative evidence generated by naturalists in the nineteenth and twentieth centuries. Deploying an innovative methodology that facilitates the transformation of the descriptive accounts of early naturalists into semi-quantitative information, the authors reconstruct and quantitatively analyze a 200-year-long time series of fish community structure indicators in the Northern Adriatic. Their findings chime with various other HMAP studies in identifying long-term changes in fish community structure, notably in this case the decline of Chondrichthyes, especially sharks, large demersals, such as hake and angler fish, and large-sized and late-maturing species like dusky grouper and brill [33].

The development of the Makassan sea cucumber (*trepang*) fishery, as traced by Kathleen Schwerdtner Máñez and Sebastian C. A. Ferse in the HMAP Collection, not only adds to HMAP's Asian case studies but also offers an example of the commercial pressures that have driven the majority of the world's fisheries over the centuries [34]. *Trepang* extraction enabled the people of Makassar, Indonesia, to profit from the export of a commodity that was in great demand in China. While this rendered them vulnerable to market fluctuations, the fishing effort was shaped by patron-client relationships and marked by the ‘roving bandit’, or bonanza, syndrome, whereby fishers exploit stocks in a locality until they are depleted, when they move to another area. The fragility of marine ecosystems in the face of seemingly rapacious human fishing activity is also the central theme of another HMAP Collection paper, Ruth H Thurstan and Callum Roberts's analysis of the ‘ecological meltdown’ that has occurred in the Firth of Clyde, Scotland, since the introduction of more intensive fishing methods in the mid-nineteenth century [35]. Previously an area that supported productive herring, cod, haddock, turbot and flounder fisheries, the impact of trawling reduced fish stocks to such a degree that the activity was prohibited in 1889. This remained so until 1962, from which point the resumption of trawling, and subsequently the deployment of ring-nets and fish finders, caused the depletion of various species, leading the authors to conclude that ‘this once diverse and highly productive environment will only be restored if closures or other protected areas are re-introduced’.

Although these studies relate to various marine species in different parts of the world, their findings not only address HMAP's key research issues, but also complement and reinforce the results of the project's initial case studies. For instance, a series of investigations into the commercial fisheries of the North Sea has revealed much about the chronology, scale and impact of the extraction of marine life from these waters over the last thousand years. Archaeological appraisals of dozens of medieval settlements showed that the period c.950–1050 saw a major rise in fish consumption around the North Sea [36]. Osteological analysis of fish bones, through their stable isotope signatures, indicates that early medieval sites are dominated by the remains of freshwater and migratory species such as eel and salmon, while later settlements reveal that the consumption of marine species such as herring, cod, hake, saithe and ling was widespread. In particular, evidence of traded cod – known as ‘stockfish’ - identified in urban areas in Norway, England, Belgium, Germany, Denmark, Sweden, Poland and Estonia, and dated at or before the mid-eleventh century, is abundant. The evidence also indicates that sea-going vessels were widely deployed by the thirteenth century to catch deep-sea fish such as ling. It is therefore apparent that substantial commercial fisheries had emerged by the eleventh century. In turn, these were a function of major economic and technological developments, as well as changes in consumption patterns that were to form the basis of dietary preferences – embracing religious practices of fasting and abstinence of red meat in favour of fish at certain weekdays and through the 40 days of Lent - which lasted into the seventeenth century.

With regard to the scale of activity, HMAP's North Sea researchers have instilled a long-term perspective into the literature. Following in the wake of Hutchings and Myers's pioneering reconstruction of catches of Atlantic cod off Newfoundland and Labrador from 1508 to 1992 [37], the first estimate of total removals of a species from the North Sea was developed for the sixteenth-century Danish inshore fisheries for herring in Scania and Bohuslen. Annual catches regularly reached a level of 35,000 tonnes [38]. By the late sixteenth century, the Dutch had taken the lead in Northern European herring fisheries with sea-going *buysen* harvesting the rich shoals off the coasts of Scotland and the Orkneys. They landed catches of 60,000–75,000 tonnes every year in the first quarter of the seventeenth century, when total removals (including English, Scottish and Norwegian landings) amounted to upwards of 100,000 tonnes. Catches declined to about half of that level by 1700, and only increased to about 200,000 tonnes in the late eighteenth century when the Swedish and Scottish fisheries developed apace. By 1870, total removals reached a level of 300,000 tonnes, which equals the Total Allowable Catch for North Sea herring in 2007, as recommended by the International Council for the Exploration of the Seas. This evidence demonstrates how fishermen in the age before steam and trawl were able to remove large quantities of biomass from the sea. While early modern catches seem to have been at a sustainable level, there are indications that removals at much lower levels than those recommended by modern standards had an effect on abundance. This can be deduced by standardizing the catching capacity of North Sea herring fishing vessels across the technological divide from sail to motor-powered vessels. Even by a conservative estimate, analysis of catch-per-unit-effort indicates that stock abundance was ten times higher in the 1600s than in the 1950s, and already by the 1800s, well before steam was introduced, it had dropped to 50–60 percent of the level of the seventeenth century. Accordingly, the impact of early modern removals of herring was much greater than historians and ecologists had previously realised [39].

A similar finding emerged from an HMAP study of the extraction of ling and cod from the North Sea. These species are classed as ‘top predators’. In ecosystem theory, top predators play a controlling and balancing role for the abundance of other species further down the food chain, and large numbers of top predators are a sure sign of healthy biodiversity. Human hunting tends to focus on top predators as the big fish are of the highest commercial value. At the same time, removing the largest specimens weakens the ecosystem, for mature fish are highly important for the reproduction of the population as their eggs are healthier and more plentiful than the spawn of younger and smaller specimens. As the fish continues to grow through its entire life, a decline in the length of specimens caught is a clear indication that fishing is changing the age structure and viability of the stock. Historical analysis demonstrated that while the average length of North Sea ling in the mid to late nineteenth century was about 1.5 metres, it had decreased to about 1.2 metres by the First World War, and ling caught today is less than 1 metre on average. A century ago, cod landed from the North Sea was usually 1-1½ metres long, while today it is only about 50 cm. This means that while cod used to live to an age of eight or ten years, in the early twenty-first century it is caught at less than three years of age. As cod only spawns at the age of three years, the fisheries are clearly removing cod at a critical stage [40].

An important aspect of any long-term perspective is the measurement of change over time. This features prominently in the contribution of Tyler D Eddy, Jonathan P.A. Gardner and Alejandro Pérez-Matus to the HMAP Collection, which focuses on the role of baselines in the management of the lobster fishery of the Juan Fernández Archipelago, Chile [41]. Having constructed baselines of lobster abundance throughout the human history of the archipelago, the authors examine the capacity of strategies such as marine reserves, effort reduction and the stewardship of catches to utilize this primary economic resource in a sustainable manner. Their findings indicate that stewardship coupled with a 30% area closure through the erection of a marine reserve would enable the stock to recover to a level midway between historic maxima and the contemporary minimum. In other words, historical evidence is being used to inform management targets and tools with the objective of rebuilding the lobster population to a user-determined size, while also providing ecosystem and biodiversity protection. This approach chimes well with the HMAP investigation into the Scotian Shelf cod fisheries, using evidence derived from the detailed log books that the skippers of fishing vessels were obliged to deposit with customs officials in order to claim a government bounty on catches. Relating to the period 1852–1866, thousands of these logbooks have been digitised and analysed to reveal that in the 1850s the adult cod biomass was in the order of 1.26 million tonnes. Remarkably, in the 1990s the comparable estimate was 50,000 tonnes. In terms of extractions, the fishermen consistently removed 200,000 tonnes of live fish per year through the 1850s. For example, in 8.5 months during 1855, the handlines used by fishermen in 43 schooners from Beverly, Massachusetts, caught just over 8,000 tonnes of cod on the Scotian Shelf, whereas in 15 months during 1999–2000 a total of just 7,200 tonnes of cod was extracted from the same waters by the entire Canadian mechanized fishing fleet, a return that fell short of the Total Allowable Catch by 11 percent [42]. This long-term comparison points to a profound change in productivity on the Scotian Shelf over the past 150 years, and a measurable reduction in abundance that is even starker than the declines of lobster in Juan Fernández, and cod and ling in the North Sea.

Like their counterparts in the Indonesian *trepang* fishery, New Englanders were aware that their prey was diminishing in extent and responded by moving to fishing grounds further offshore. By the late 1850s, many schooners were undertaking longer voyages to the Gulf of St Lawrence and the Grand Banks, where stocks were perceived to be larger. Another response, which was also evident contemporaneously in the Firth of Clyde, was the application of new technology. French fishermen introduced tub trawls to the Scotian Shelf fishery, and soon the Americans no longer used the traditional handlines with 2–4 hooks per man, but longlines of upwards of 400–500 hooks per crewman. While the catchment area of one boat increased immensely, and catches went up in the short run, in a matter of a few years the fish stock was showing clear depletion signals, with smaller individuals being caught and the catch-per-unit-effort of fishermen declining [43]. In essence, these New England fishermen were interacting with the marine environment in ways that were not only evident in earlier historical settings, but have also become very familiar since the 1850s: faced with environmental changes, which their activity had precipitated, they extended the spatial scope, and enhanced the intensity, of their fishing effort.

Spatial range is also a key theme of the research undertaken as part of the HMAP World Whaling case study by Tim Smith, Randall Reeves, Elizabeth Josephson and Judith Lund. This team has analyzed data relating to American offshore whaling voyages to describe the historical distribution of five key groups of species that were targeted by nineteenth-century whalers: sperm, right, humpback, gray and bowhead whales. The data are presented in the form of world maps, showing where the whalers went and where they encountered these species of whales [44], and will be described in detail in a paper planned for the HMAP Collection. Comparing these distributions with what is known of the present-day distribution of these species identifies areas where whales do not appear to inhabit their historical ranges, suggesting that comparisons of past and current ranges should be given greater consideration in the management of whales today. This work builds upon a body of research outputs generated by the team. In the early stages of the project, they attempted to identify all of the world's whale fisheries, from aboriginal harpoon fisheries with origins in antiquity to shore-based commercial fisheries, and finally to high seas commercial fisheries beginning before the nineteenth century and continuing today [45]. Noting that the twentieth-century catches of the great whales were relatively well known [46], the team focused most of their effort on the nineteenth century, when the main offshore whaling nations were the United States, Britain and France, with the American fishery being far and away the largest and best documented. The team assembled summary data on all recorded American offshore whaling voyages [47], which totalled more than 15,000, primarily in the eighteenth and nineteenth centuries. They also extracted data from a sample of voyage logbooks kept by American whalers, and rescued earlier data that had been extracted from some of these logbooks in a study in the 1850s and another in the 1930s. These data provide detailed spatial information on where whalers went and on the numbers of whales taken on each sampled voyage.

The team used these offshore whaling voyage data, as well as other archival sources from shore-based whaling operations, to develop more detailed descriptions for several areas of the magnitude of whaling, and its impact on for four key nineteenth-century target whales: right, sperm, gray and humpback. Right whales were the earliest target species, beginning at least by 1050 AD and continuing in the North Atlantic in some 33 fisheries for over 1000 years. Right whales were pursued in all the world's oceans, both by shore-based and offshore whalers. Total removals of right whales in the western North Atlantic were estimated to have been at least 5,000 animals [48], far more than the current population of several hundred animals, while roughly 25,000 right whales were taken from New Zealand waters in the 1800s [49]. In the North Pacific, the team demonstrated that rapid spatial shifts in right whaling occurred over the decade of the 1840s and resulted in a swift decline in the rate at which whalers encountered right whales [50]. The idea that the right whales were at one time distributed broadly across the North Pacific was shown to be wrong, with the highest encounter rates occurring east of 160 deg W and west of 170 deg E [51].

The other major target of nineteenth-century whalers were sperm whales. The team drew on published and archival sources to identify more that 60 sperm whaling grounds [52], and also addressed an apparent inconsistency between order of magnitude declines in nineteenth-century sperm whale encounter rates [53], [54] and the current status of this species globally, estimated at 70% of pre-whaling abundance [55]. This latter study was based on estimates of current global abundance and estimated catches in the eighteenth, nineteenth and twentieth centuries of over one million animals. The team suggested that this inconsistency is in fact most apparent in the North Pacific, and hypothesized that the region north of 40 deg N latitude may have been a refuge for sperm whales during the nineteenth century, a refuge that was breached in the twentieth century [56]. While it is apparent that sperm whale abundance declined in the first half of the eighteenth century in at least the North Pacific, it is less clear if this was a major contributor to the eventual decline of American whaling. The team demonstrated the limitations of global analyses of sperm whaling, and used regional analyses to show that the effect of whaling on sperm whales may have differed substantially between the Pacific and the Atlantic [57]. Over the first half of the nineteenth century, rates of encounter of sperm whales did not decline in the Atlantic as they had in the Pacific, and by the second half of the nineteenth century American whalers had retreated from the Pacific back into the Atlantic. Determining the causes of the decline of American whaling is complicated by the complex spatial changes in whales and whaling.

Humpback whales have been sought in the North Atlantic since the seventeenth century, with at least one fishery continuing to the present, albeit at very low levels. Both shore and offshore whalers pursued this species on its two North Atlantic breeding grounds and in all of its many feeding grounds. The team examined all archival information that it could find and developed estimates of total removals of around 30,000 animals [58]. The number of humpback whales alive before whaling (pre-whaling abundance) was estimated using population models based on estimates of removal and present-day abundance to be between 21,000 and 24,000 whales [59], [60]. This number is an order of magnitude lower than estimates of average long-term abundance estimated from genetic variability [61]. The cause of this discrepancy is under investigation.

Extinct in the North Atlantic in the 1600s, gray whales became a target of whaling in the North Pacific, being pursued for several centuries in both their western and eastern North Pacific populations. In the eastern North Pacific, gray whaling was long conducted aboriginally on well-defined migration and feeding grounds. In the 1850s, commercial whalers from several nations began to focus on this species in its calving and breeding grounds in Baja California and in the North Pacific feeding grounds. American shore-based whaling also developed along the California coast. Although the total removals of eastern North Pacific (or California) gray whales had previously been estimated, those estimates were inconsistent with sightings-based estimates of current and recent abundance, and as a result pre-whaling abundance has been poorly understood. The World Whaling team revisited the estimates of nineteenth-century gray whaling in the eastern North Pacific to determine if the source of this inconsistency was biases in estimates of removals [62], [63]. Deploying substantially different methods than used previously, their new estimates were remarkably similar to the earlier estimates. Additional information is becoming available in the form of genetic based estimates of long-term average abundance for both the eastern and western North Pacific populations taken together [64] and improved estimates of present day abundance [65]. Work is continuing to determine pre-whaling abundance.

The HMAP Baltic case study has shed much light on the historical development of fisheries in the region. Over the long term, little pressure was exerted by commercial fishing on fish stocks in the inner parts of the Baltic. During the late seventeenth century, for example, removals of fish biomass from the Gulf of Riga were at least 200 times less than the level they reached in the late twentieth century. In the earlier period, moreover, the bulk of the fishing effort was expended in the rivers. Migratory fish species, such as sturgeon, Atlantic salmon, brown trout, whitefish, vimba bream, smelt, eel and lamprey were the most important commercial fish in the area, because they were abundant, had high commercial value and were easily available. Over time, however, fishing activity moved downstream and into the sea. Due to intensive fishing, populations of many migratory species, especially sturgeon and Atlantic salmon, contracted considerably and they became less commercially significant, while marine fish, especially Baltic herring, increased in importance during the nineteenth century [66]. In a paper to be published in this HMAP Collection, Brian MacKenzie, Margit Eero and Henn Ojaveer focus on the relationship between predators and prey to project whether the cod stock can recover if seals also recover [67]. In so doing, they refer to the experience of earlier centuries, for which the bulk of the evidence indicates that the two species were present in some abundance. But this does not necessarily mean that the same situation will occur in the future, for other variables, most notably fishing pressure and climatic conditions, may well have changed. Drawing a schematic of the upper trophic levels of the Baltic foodweb in different centuries, and applying population modelling techniques, the authors provide research-informed advice for resource management agencies.

This follows an established pattern, for the HMAP Baltic team has utilized long-term perspectives to help solve other environmental issues. For instance, in the absence of historical records before 1966, fishery managers asked if the record high cod stock in the Baltic Sea in the late 1970s and early 1980s was a unique occurrence, or whether it was likely to happen at regular intervals. The question was unequivocally answered through the recovery of historical data back to 1925, which showed that abundant cod stocks corresponded to a favourable combination of four key drivers: incursions of saline water to the brackish Baltic and hydrographic conditions that facilitated successful reproduction; low marine mammal predation; a highly productive environment fuelled by nutrient loading; and reduced fishing pressure. Such a conjunction of factors did not take place at any other point in the twentieth century. While the cod biomass was restricted from 1920 to 1950 by an abundance of marine mammals and low ecosystem productivity, in the 1950s and 1960s stock levels were depressed by high fishing pressure, and hydrographic conditions were rarely conducive to good reproduction rates throughout the twentieth century, especially after 1985. The late 1970s and early 1980s were therefore extraordinary in that a combination of positive factors interacted to produce a large cod stock, a conclusion that will perhaps inform the policies and targets of fisheries managers [68].

A further notable finding of HMAP Baltic research relates to the resilience of fish to broad changes in temperature and other meteorological variables. Archaeological evidence of fish fauna in the Atlantic warm period (c.7000-3900 BC) infers that there were many fish species in the waters around Denmark which are now be found in warmer waters. However, cod was very abundant in the Stone Age, even though temperatures were 2–4 degrees warmer those of the late twentieth century, suggesting that significant cod populations can be maintained in the Baltic region even if temperatures rise due to global warming, provided that fishing mortalities are reduced. Climatic variables also influenced the abundance and distribution of other species. For instance, during the Little Ice Age of the late seventeenth century, cold-water marine fish (herring, flounder and eelpout) sustained important fisheries in the Baltic, while the fishing season for the major pelagic fish species was much later in the year, compared to the much warmer conditions of the present day. Similarly, the magnitude and composition of catches of herring and other coastal fish (e.g. perch and ide) near Estonia in the mid and late nineteenth century, when fishing effort and methods were constant, were chiefly governed by climatic fluctuations [69]. The influence of another natural factor, the quality of the water, has also been highlighted by historical analysis of the hydrographic event that ensued when the North Sea breached the fragile coast of the Limfjord in 1825. In this instance, the saltwater intrusion destroyed the habitat for freshwater whitefish and created conditions that favoured saltwater species such as plaice – an environmental shock that drastically altered the character of the human fishing effort in this area [70].

### A short view on the long-term perspective

A decade ago, the editors of the first collection of HMAP research papers anticipated that the findings of the project's initial case studies would make ‘a major contribution to knowledge and understanding of the complex, delicate and important relationship between human societies and the marine environment’ [31]. We can now report that the multidisciplinary approach fostered by HMAP has generated a substantial corpus of work that offers long-term perspectives on changes in stock abundance, the ecological impact of large-scale human harvesting and the role of marine resource utilization in the development of human societies. Such a view, in turn, broadens and deepens knowledge of the contemporary condition of the marine environment and provides the time series and ecological insight required to assess the future sustainability of marine animal populations. We are confident that the papers in this Collection – those currently available (as of December 2010) and those to be added subsequently - will augment and enhance the HMAP contribution to historical marine ecology and marine environmental history.
